The article "Feasibility and Efficacy of a Degradable Magnesium-Alloy GBR Membrane for Bone Augmentation in a Distal Bone-Defect Model in Beagle Dogs" was published in 2022. Journal: Bioinorg Chem Appl.

# Feasibility and Efficacy of a Degradable Magnesium-Alloy GBR Membrane for Bone Augmentation in a Distal Bone-Defect Model in Beagle Dogs

**DOI:** 10.1155/2022/4941635

**Published:** 2022-03-23

**Authors:** Zi-Yu Yan, Jian-Hua Zhu, Guan-Qi Liu, Zhi-Chao Liu, Chuan-Bin Guo, Nian-Hui Cui, Jian-Min Han

**Affiliations:** ^1^Department of Oral and Maxillofacial Surgery, Peking University School and Hospital of Stomatology, Beijing, China; ^2^National Engineering Laboratory for Digital and Material Technology of Stomatology, Department of Dental Materials, Peking University School and Hospital of Stomatology, Beijing, China; ^3^School of Materials Science and Engineering, Beijing Institute of Technology, Beijing, China

## Abstract

We explored the feasibility and efficacy of a degradable magnesium (Mg) alloy guided bone regeneration (GBR) in the treatment of bone defects after tooth extraction. A GBR membrane (MAR-Gide (MG)) was used to treat a mandibular second molar (M2M)-distal bone defect (DBD). In eight beagle dogs, bilateral mandibular second and fourth premolars were hemi-sected. The distal roots were removed to create a two-wall bony defect of dimension 5 mm × 5 mm × 5 mm to simulate M2M-DBD. Thirty-two bone defects were assigned randomly into four groups according to GBR membranes (MG and Bio-Gide (BG)) applied and the time of killing (3 months and 6 months after surgery). The osteogenesis of bone defects and MG degradation were analyzed using micro-CT, histology (staining, tartrate-resistant acid phosphatase), and inductively coupled plasma mass spectrometry. MG did not increase the prevalence of infection, wound dehiscence, or subcutaneous emphysema compared with those using BG. Trabecular volume/total volume at 3 months (63.71 ± 10.4% *vs*. 59.97 ± 8.94%) was significantly higher in the group MG than that in the group BG. Implanted MG was degraded completely within 3 months, and “island-shaped” new bone was found near MG degradation products. A significant difference was not found in vertical bone height or percent of new bone formation (45.44 ± 12.28% *vs*. 43.49 ± 7.12%) between the groups. The concentration of rare-earth elements in mandibular lymph nodes of the group MG was significantly higher than that of the group BG (*P* ≤ 0.017) but did not lead to histopathological changes. In summary, MG exhibited good biocompatibility and clinical applicability compared with BG in vivo. The osteogenic effect of MG could be enhanced by regulating the degradation rate of Mg-alloy.

## 1. Introduction

The distal bone defect (DBD) of the mandibular second molar (M2M) is a common complication after M3M extraction. Kugelberg et al. followed the fate of M2M distal periodontal tissue after M3M extraction for 2 years. They found that the probing depth exceeded 7 mm in 43.3% of cases and that 32.1% of bone defects exceeded 4 mm [1]. Deep periodontal pockets create a local anaerobic environment, which is conducive to the growth of pathogenic bacteria and may, ultimately, affect the long-term preservation of teeth [2, 3].

The article "Feasibility and Efficacy of a Degradable Magnesium-Alloy GBR Membrane for Bone Augmentation in a Distal Bone-Defect Model in Beagle Dogs" was published in 2022. Journal: Bioinorg Chem Appl.

The treatment of M2M-DBD is a challenge for oral surgeons. Guided bone regeneration (GBR) is an efficacious treatment for most bone defects after tooth extraction [4]. GBR promotes bone augmentation if barrier membranes are employed to prevent non-osteogenic tissue from growing into bone defect sites. However, GBR is not always efficacious against M2M-DBD because most membranes cannot cope with the complicated bone defect at this site [5, 6]. First, M2M-DBD is large and requires the barrier membrane to have a certain mechanical strength to maintain space during osteogenesis. Besides, the retro-molar region lacks keratinized gingiva [7], so infection and secondary surgical trauma have considerable influence upon M2M-DBD healing. However, neither absorbable membranes (e.g., collagen membrane) nor nonabsorbable membranes (e.g., titanium mesh or polytetrafluoroethylene) used commonly can meet the requirements for M2M-DBD treatment stated above. A collagen membrane cannot maintain the osteogenesis space. Titanium mesh increases the risk of infection and secondary surgical trauma to the operated area. The effect of GBR is closely related to the characteristics of barrier membranes [6, 8]. Finding new GBR membranes that possess good mechanical properties, antibacterial properties, and absorbability to improve the prognosis of M2M-DBD is important.

Degradable magnesium (Mg)-alloys are “ideal” biological materials for GBR membranes due to their excellent properties. Mg-alloys have good biocompatibility [9, 10]. Many biological products made of Mg-alloys, such as vascular stents and orthopedic screws, have been applied clinically and achieved good results [11, 12]. The mechanical properties of Mg-alloys can maintain the osteogenesis space, which is important for M2M-DBD where vertical ridges augmentation is required [13]. The elastic modulus of Mg-alloys is similar to that of natural bone [14]. Hence, Mg-alloys can reduce the stress shielding effect and reduce the risk of membrane exposure compared with that using titanium mesh [14, 15]. After processing into a membrane for GBR, trimming and bending them to adapt to the complex shape of the defect is easy due to their good plasticity [16]. In addition, the degradability and antibacterial properties of Mg-alloys can reduce the risk of infection and secondary surgical trauma to the fragile keratinized gingiva at M2M-DBD [7, 17]. Moreover, magnesium ions (Mg^2+^) can further promote bone repair by regulating signal transduction between osteoblast-related cells [9]. Mg-alloy GBR membranes with excellent properties are expected to improve the prognosis of M2M-DBD.

The article "Feasibility and Efficacy of a Degradable Magnesium-Alloy GBR Membrane for Bone Augmentation in a Distal Bone-Defect Model in Beagle Dogs" was published in 2022. Journal: Bioinorg Chem Appl.

Reports on the clinical application of Mg-alloy GBR membranes are lacking. The main difficulty in the clinical application of Mg-alloy biomaterials is the regulation of their degradation rate. Uncontrolled degradation of Mg-alloys leads to rapid release of hydrogen and affects their biological functions (e.g., biocompatibility, osteogenesis, and antibacterial) [18]. The key problem that needs to be solved in the development of Mg-alloy GBR membranes is to control their degradation rate to adapt to bone healing.

The magnesium-zinc-yttrium-neodymium (Mg-Zn-Y-Nd) alloy developed by our research team has improved its corrosion and mechanical properties [19]. The content of rare-earth elements (REEs) in Mg-Zn-Y-Nd alloy is only one-third of that of magnesium electron WE43 (a Mg-alloy used commonly in medicine), which indicates that it has greater biological safety [20]. In addition, we have used Mg-alloy GBR membranes to repair skull defects in rats and demonstrated its good biocompatibility and osteogenic effect [21].

We further improved the corrosion resistance of the Mg-alloy by fluorination treatment and intended to use it to repair a complicated bone defect such as M2M-DBD. A M2M-DBD model was created based on the mandibles of beagle dogs, which could better reflect the clinical application of a GBR membrane and lead to a clinically instructive conclusion. We aimed to explore the therapeutic effect of a Mg-alloy on the treatment of a complicated bone defect as well as its degradation rate and osteogenesis.

## 2. Methods

### 2.1. Ethical Approval of the Study Protocol

The ethics committee of Peking University Hospital of Stomatology (Beijing, China) approved the research protocol (LA2018008). All procedures were undertaken according to Animal Research: Reporting of In Vivo Experiments (ARRIVE) guidelines.

### 2.2. Sample Preparation

Each degradable Mg-alloy regeneration membrane (MAR-Gide (MG)) applied in this study was processed from an extruded Mg-2Zn-0.46Y-0.5Nd (wt%) alloy bar as the substrate [19], which was provided by Materials Research Center in Zhengzhou University (Zhengzhou, China). According to the characteristics of M2M-DBD, the bar was cut into disks of thickness 150–200 *μ*m by a wire electrode. After grinding and polishing, these disks were processed to an appropriate shape by cutting with a microsecond laser. Some holes were designed on the membrane. The large holes (1.2 mm in diameter) were used for fixation of Mg-alloy nails, whereas the small holes (0.5 mm in diameter) were designed for nutrition supply (Figure 1(e)). The disks were washed ultrasonically for fluorination treatment. First, all samples were treated in boiled NaOH solution (1 mol/L) for 2–6 h. Then, they were reacted with hydrofluoric acid (HF) solution (20 wt%) for 2–6 h at room temperature to fabricate a uniform magnesium fluoride (MgF2) layer on the substrate surface. Finally, the MGs were sterilized by *γ*-rays for 30 min on each side and were ready for use. In addition, the Mg-alloy nails (length = 3 mm; diameter = 1 mm; and head diameter = 3 mm) used for fixation was also developed by our research team. They were also processed with Mg-2Zn-0.46Y-0.5Nd (wt%) alloy and fluorinated in a similar way to MG.

The article "Feasibility and Efficacy of a Degradable Magnesium-Alloy GBR Membrane for Bone Augmentation in a Distal Bone-Defect Model in Beagle Dogs" was published in 2022. Journal: Bioinorg Chem Appl.

### 2.3. Microstructure and Compositional Analysis of MGs

A field emission scanning electron microscope (S8230; Regulus, Tokyo, Japan) in second-electron mode with an energy-dispersive spectrometer was used to characterize the microstructure and element mapping of the surface and cross section of MGs. The acceleration voltage and working distance were set to 15 kV and 15 mm, respectively. X-ray photoelectron spectroscopy (XPS) using a PHI Quantera II SXM system (ULVAC-PHI, Kanagawa, Japan) was employed to characterize the surface chemical state of samples with Al K *α* radiation (1486.6 eV) as the excitation source to record the data. The spectral charge was corrected with the binding energy of the C1s signal. The Shirley method was carried out for background subtraction of all spectra. The survey spectrum and high-resolution spectra for the Mg2p signal were imported to MultiPak (ULVAC-PHI) involving Gaussian multi-peak fitting for further analyses.

### 2.4. In Vivo MG Implant

A split-mouth randomized controlled trial was designed according to the work of Ge et al. [13]. Eight healthy beagle dogs (1–1.5 years; average weight = 15 kg) were used. For each beagle dog, bilateral mandibular P2 and P4 were hemi-sected and made to simulate M2M-DBD. Thirty-two bone defects were assigned randomly into four groups with eight sites in each group: I was MG-3 months (MG-3 m); II was Bio-Gide-3 months (BG-3 m); III was MG-6 m; and IV was BG-6 m. Beagle dogs were killed 3 months after surgery in groups I and III and 6 months after surgery in groups II and IV.

Beagle dogs were anesthetized (3% pentobarbital sodium (30 mg/kg), i.m.). The surgical area was disinfected with 0.5% povidone iodine. Local anesthesia was induced with 2% lidocaine before surgery. Full-thickness mucoperiosteal flaps were elevated and bilateral mandibular P2 and P4 were hemi-sected. Distal roots were removed, and the canals of the mesial roots were reamed and filled with iRoot® SP (Innovative BioCeramix, Vancouver, Canada) (Figures 1(a) and 1(b)). Subsequently, the extracted distal root was processed to an autologous fresh dentin matrix (DM). The enamel, pulp, cementum, and fibrous tissue were removed first. Then, the teeth were ground to particles of diameter ∼500 *μ*m with a bone grinder (Kohler, Lahr/Schwarzwald, Germany) and cleaned with sterile phosphate-buffered saline before grafting.

The article "Feasibility and Efficacy of a Degradable Magnesium-Alloy GBR Membrane for Bone Augmentation in a Distal Bone-Defect Model in Beagle Dogs" was published in 2022. Journal: Bioinorg Chem Appl.

The mesial and buccal bone walls of the extraction sockets were removed surgically to create a two-wall bony defect of dimension 5 mm × 5 mm × 5 mm (Figures 1(c) and 1(d)). After grafting the DM into the bone defect, MG and BG (Geistlich Pharma North America, Princeton, NJ, USA) were trimmed and covered on the surface according to the study design. MG was fixed with Mg-alloy nails (Figures 1(f)–1(h)). The flaps were closed after tension reduction. All surgical sites were protected with periodontal dressing materials (Figure 1(i)).

Penicillin (30,000 units/kg bodyweight, i.m.) was administered for 3 days. Soft food was provided for the first week after surgery. Clinical follow-up was done regularly after surgery. The beagle dogs were killed after 3 months or 6 months with an overdose of 3% pentobarbital sodium. The remaining mesial root, bone defect, and related mucosa were harvested. Samples were fixed in 10% neutral formalin and prepared for micro-computed tomography (CT) and histology. The submandibular lymph nodes were also dissected. The number and size of lymph nodes were recorded. Then, each lymph node was sectioned longitudinally into two pieces: one for analyses of MG-related elements, and the other was fixed in 10% neutral formalin and prepared for histology.

### 2.5. Micro-CT

A multi-modality Micro-CT scanner (80 kV, 500 *μ*Ad. Micro-CT data were imported into Inveon Research Workplace 4.2 for further analyses. The M2M-DBD was extended from the distal aspect of M2M, so the region of interest (ROI) was set according to the bone-defect model (dimension 5 mm × 5 mm × 5 mm) to represent regenerated bone. The trabecular area was determined using a Gaussian filter (sigma = 0.8; threshold = 22%). Referring to the histological features of identical sites, the bone density-like film image was considered to be a suspected Mg residual. The average bone mineral density (BMD), percent trabecular area (trabecular volume/total volume of ROI (BV/TV)), trabecular thickness (Tb. Th), trabecular number (Tb. N), trabecular separation (Tb. Sp), and vertical bone height (VBH) were calculated using Inveon Research Workplace 4.2. The VBH was recorded as the linear distance from the enamel-cementum junction to the bottom of the bone defect (Figure 2).

The article "Feasibility and Efficacy of a Degradable Magnesium-Alloy GBR Membrane for Bone Augmentation in a Distal Bone-Defect Model in Beagle Dogs" was published in 2022. Journal: Bioinorg Chem Appl.

### 2.6. Histology

Bone-defect blocks were divided randomly into two parts. One portion of bone-deflect blocks (3/8 samples) was decalcified (10% EDTA-2Na and agitation in a 37°C water bath shaker), dehydrated (in an ascending series of ethyl alcohol concentrations from 70% to 100%), and embedded in paraffin. Sagittal sections of thickness 5 *μ*m were cut and stained with hematoxylin/eosin (H&E) and tartrate-resistant acid phosphatase (TRAP). Images were captured under a light microscope (CKX-41; Olympus, Tokyo, Japan) with a charge-coupled device camera. The number of TRAP (+) cells was evaluated quantitatively under field of views of magnification 200x. Three views in the bone defect area were selected randomly. The average number of TRAP (+) cells was defined as the number of osteoclasts.

The other portion of bone-defect blocks (5/8 samples) was dehydrated and embedded in polymethyl methacrylate resin (Wako Pure Chemical Industries, Tokyo, Japan). At the center of each block, sections of size 300 *μ*m were cut using a diamond saw (STX-202A; Shenyang Kejing Auto-instruments, Liaoning, China). Then, they were ground and polished to a thickness of 50 *μ*m. These non-decalcified sections were stained (Van Gieson's) and observed under a light microscope. MG degradation and the response of surrounding tissues were observed. Percentage new bone formation (% NBF) was determined using ImageJ (US National Institutes of Health, Bethesda, MD, USA). In addition, half of each mandibular lymph node was dehydrated, embedded, and stained with H&E for observation under a light microscope.

### 2.7. Analyses of MG-Related Elements in Lymph Nodes

Each submandibular lymph node was cut along the long axis and divided into two portions. One portion was made into sections and stained with H&E for histological observation of inflammation, hemorrhage, and necrosis. The other portion was weighed accurately and digested with nitric acid: perchloric acid (9 : 1) in a microwave oven. Later, ultrapure water was applied to replace this acid mixture. The concentration of each element (Mg, Zn, Y, and Nd) was determined by inductively coupled plasma mass spectrometry (Thermo Scientific, Waltham, MA, USA). The standard for each element was provided by China Metrology Science Research (Beijing, China) and the National Nonferrous Metals and Electronic Materials Analysis and Testing Center (Beijing, China).

### 2.8. Statistical Analyses

Data were analyzed using SPSS 21.0 (IBM, Armonk, NY, USA) and are presented as the mean ± standard deviation. The chi-squared test, paired *t*-test, independent *t*-test, and nonparametric analysis were applied. *P* < 0.05 was considered significant.

The article "Feasibility and Efficacy of a Degradable Magnesium-Alloy GBR Membrane for Bone Augmentation in a Distal Bone-Defect Model in Beagle Dogs" was published in 2022. Journal: Bioinorg Chem Appl.

## 3. Results

### 3.1. Microstructure and Composition of MG

According to observation of the surface and cross section of MG, the fluorinated film was uniform with a thickness of ∼3 *μ*m (Figure 3). Scanning electron microscopy images revealed the surface coating of MG to be uniform. Cracks (width <0.2 *μ*m) were distributed uniformly on the surface. Energy-dispersive spectrometry mapping showed some particles composed of REEs to be scattered partially on the surface.

XPS showed the surface of MG to be coated mainly with MgF_2_ and Mg (OH)_2_. The high-resolution spectrum of Mg2p is shown in Figure 4(a). According to the standard database [22], the spectrum could be resolved into two components: a major one at 51.50 eV corresponding to MgF_2_ and a minor one at 50.50 eV corresponding to Mg (OH)_2_. The atomic ratio of F : Mg was ∼2 : 1 (46.93% *vs*. 21.58%) (Figure 4(b)).

### 3.2. Clinical Evaluation

There was no significant difference in the prevalence of membrane exposure, wound dehiscence, infection, or subcutaneous emphysema between the group MG (*n* = 16) and group BG (*n* = 16). Two sites in the group MG and one site in the group BG were infected. One site in the group MG was found to be exposed 4 days after surgery. The membrane was broken and peeled off partially, accompanied by local wound dehiscence. Another site in the group MG was found to be infected 3 months after surgery. Interestingly, the corresponding contralateral site in the group BG was also infected. Those two sites were in the P2 region. The remaining mesial roots were found to have roots broken and the mobility of them were degree III. All other sites healed normally without obvious complications. Subcutaneous emphysema was not found in the group MG.

There was no difference in the size and number of lymph nodes between the group MG and group BG. The lymph nodes were about 0.5–1 cm in diameter, with good mobility and clear borders. Visually enlarged or necrotic lymph nodes were not found in either group.

### 3.3. Micro-CT

Micro-CT revealed the speed of bone repair in the group MG to be faster than that in the group BG. The value of BV/TV in group MG-3 m was significantly higher than that in the group BG-3 m (63.71 ± 10.4% *vs*. 59.97 ± 8.94%, *P*=0.050). Compared with the group BG-3 m, the trabecular bone in the group MA-3 m was thinner (Tb. Th: 0.45 ± 0.11 *vs*. 0.52 ± 0.12 *μ*m, *P*=0.001), denser in separation (Tb. S: 0.25 ± 0.07 *vs*. 0.35 ± 0.1 *μ*m, *P*=0.001), and greater in number (Tb. N: 1.45 ± 0.2 *vs*. 1.19 ± 0.22/mm, *P* < 0.001). However, 6 months after surgery, no difference was found between the values of BV/TV in the group MG-6 m and group BG-6 m. From 3 months (group MG-3 m) to 6 months (group MG-6 m) after surgery, the density and thickness of bone increased, whereas the number of new bones decreased, but these changes were not significant. No significant difference was found in the VBH between the group MG and group BG (3 months: 2.83 ± 0.62 *vs*. 3.38 ± 0.99 mm, *P*=0.084; 6 months: 2.87 ± 0.54 *vs*. 2.75 ± 0.92 mm, *P*=0.704) (Figure 5). Imaging of suspicious residual MG material was not found in the group MG.

The article "Feasibility and Efficacy of a Degradable Magnesium-Alloy GBR Membrane for Bone Augmentation in a Distal Bone-Defect Model in Beagle Dogs" was published in 2022. Journal: Bioinorg Chem Appl.

### 3.4. Histology

Initially, the rate of bone regeneration in the group MG was higher than that in the group BG, but a significant difference was not found over the long term between these two groups. Repair of new bone could be observed clearly in the group MA-3 m, whereas the defect area in the group BG-3 m was filled with more fibrous connective tissue (Figures 6(a) and 6(b)). Percent NBF in the group MG-3 m was higher than that in the group BG-3 m (51.64 ± 12.77% *vs*. 39.99 ± 5.95%, *P*=0.257). However, multinucleated TRAP (+) cells were observed along the bone-defect margin. The number of TRAP (+) cells per field of view at 200x magnification was significantly higher in the group MG than that in the group BG (3.73 ± 1.5 *vs*. 2.13 ± 1.15, *P*=0.035) (Figures 6(c)–6(f)). The increase in the vertical height of distal bone defect was limited, and an obvious difference between the two groups was not observed. In general, %NBF in the group MG was similar to that in the group BG (45.44 ± 12.28% *vs*. 43.49 ± 7.12%, *P*=0.704). Severe inflammation or tissue necrosis was not found in the group MG or group BG.

New bone was observed to originate from the margin of the bone defect in both groups. However, “island-shaped” new bone was found only in the group MG. Residual MG was not found in the bone defect area, but some degraded particles of MG were found in the group MG-3 m, which were “swallowed up” by monocytes (400x magnification). Interestingly, island-shaped new bone was formed accompanied by the degradation products of MG (Figures 7(a)–7(f)). Degraded particles of MG were not found in the group MG-6 m. In addition, gas cavities were found in only one section of the group M0047-3 m. These gas cavities were divided into compartments surrounded by fibrotic tissue (Figures 7(g) and 7(h)). DM particles were almost completely absorbed or remodeled. Only a very small amount of the DM was observed in some sections.

An abnormality in the histological structure of the lymph nodes was not found in the group MG or group BG. The cortex and medulla of lymph nodes were demarcated clearly, and the cortex was thin and uniform. Lymphoid nodules with clear outlines could be found within lymph nodes. Pathological changes (e.g., bleeding, local necrosis) were not found.

The article "Feasibility and Efficacy of a Degradable Magnesium-Alloy GBR Membrane for Bone Augmentation in a Distal Bone-Defect Model in Beagle Dogs" was published in 2022. Journal: Bioinorg Chem Appl.

### 3.5. MG-Related Elements in Lymph Nodes

REEs were metabolized slowly through lymphatic circulation, but they accumulated in the submandibular lymph nodes in the group MG. The concentration of REEs (*μ*g/L) in the group MG was significantly higher than that in the group BG (Y: 0.35 ± 0.55 *vs*. 0.01 ± 0.05, *P*=0.014; Nd: 1.00 ± 1.60 *vs*. 0.05 ± 0.16, *P*=0.017). The content of Y and Nd (in *μ*g/L) was higher in the group MA-6 m than that in the group MA-3 m (Y: 0.56 ± 0.66 *vs*. 0.14 ± 0.34, *P*=0.394; Nd: 1.62 ± 1.97 *vs*. 0.39 ± 0.91, *P*=0.240). However, the content of Y and Nd (in *μ*g/L) decreased in the group BG (group BG-3 m *vs*. group BG-6 m : Y: 0.03 ± 0.07 *vs*. 0, *P*=0.699; Nd: 0.09 ± 0.22 *vs*. 0.01 ± 0.01, *P*=0.699) (Figures 8(g) and 8(h)).

A significant difference was not observed in the concentration (in *μ*g/L) of Mg (98.71 ± 19.71 *vs*. 109.04 ± 33.11, *P*=0.443) or Zn (6.98 ± 3.16 *vs*. 8.61 ± 1.51, *P*=0.242) between the group MG and group BG (Figures 8(e) and 8(f)).

## 4. Discussion

We attempted to apply an Mg-alloy GBR membrane to promote bone healing of complicated bone defects (M2M-DBD model in beagle dogs) and explored the coordination of degradation of Mg-alloy and osteogenesis. The MG used in our study exhibited good clinical applicability and biocompatibility compared with that of BG in vivo. MG had the potential of osteoinduction, and its osteogenic effect was not inferior to that of BG. MG could degrade completely within 3 months after surgery without leading to subcutaneous emphysema or increasing the infection risk compared with that using BG. The osteogenic effect of MG could be enhanced further by regulating the degradation rate of Mg-alloy. We demonstrated, for the first time, that MG could promote bone healing in mandibular bone defects.

The key to MG application in the oral cavity is exploration of its degradation rate, which can be adapted to the bone repair process and ensure the biological safety of the material simultaneously. The bone healing-promoting effect of the Mg-alloy on bone defects is manifested macroscopically and microscopically. Macroscopically, the Mg-alloy can maintain the osteogenesis space during osteogenesis, which is critical to the osteogenesis effect of GBR technology [4]. The Mg-alloy can also degrade slowly in vivo, which reduces the impact of secondary surgical trauma upon osteogenesis [11, 12]. Microscopically, the Mg-alloy and its degradation products can affect the local microenvironment and exert its biological properties (e.g., antibacterial, bone-promoting) [9, 17]. However, to achieve such functions, control of the degradation rate of the material is needed. The biological safety of materials is also closely related to the rate of degradation. Uncontrolled degradation of Mg-based materials can cause subcutaneous emphysema, wound dehiscence, and infection [18]. Therefore, regulation of the degradation rate of MG is crucial for its clinical application.

The article "Feasibility and Efficacy of a Degradable Magnesium-Alloy GBR Membrane for Bone Augmentation in a Distal Bone-Defect Model in Beagle Dogs" was published in 2022. Journal: Bioinorg Chem Appl.

The degradation rate of MG used in the present study was regulated effectively after anticorrosion treatment. Alloying with other elements and surface modification are the most commonly used methods to control the degradation rate [23]. After alloying with REEs, the Mg-Zn-Y-Nd alloy used in our study not only improved its anticorrosion resistance, but also maintained its good biocompatibility and clinical applicability, which has been demonstrated in various in vitro and in vivo studies [24–26]. In addition, there was a uniform coating on the surface of the material, the main components of which were MgF_2_ and Mg (OH)_2_ (Figures 3 and 4). HF treatment can elicit surface passivation to control the degradation rate [16, 27]. MgF_2_, oxides, and Mg (OH) xF_2_–x can form on the surface of Mg-alloys, and the corrosion rate has been shown to be 20-fold lower than that of untreated samples [16, 27]. The ability of similar fluorinated films to improve the anticorrosion resistance of the substrate has been demonstrated [28–30].

MG could promote bone healing in our M2M-DBD model. BV/TV and %NBF in the group MG-3 m were greater than those in the group BG-3 m (Figure 6). The most likely explanation for this phenomenon is that MG promoted osteogenesis through its mechanical properties and local degradation. Residual MG was not observed in the group MA-6 m, but some degradation particles of Mg-alloy were observed by histology in the group MA-3 m (Figure 7), which indicated that MG could maintain its mechanical strength for a period of time and degraded completely within 3 months in vivo. In addition, the formation of new bone was found not only from the margin of the bone defect, but also close to the degradation products of MG (Figure 7), which indicated that MG had the potential for osteoinduction [31, 32]. Micro-CT results confirmed our assumptions. The new bone was more porous in the group MG than that in the group BG, and the trabecular separation decreased gradually in the group MG (Figure 5). These observations were consistent with those of our previous study [21], indicating that many isolated bone islands were formed initially and then fused gradually in the group MG. Qiao et al. reported that administration of an appropriate amount of Mg^2+^ in the early stage of inflammation could stimulate macrophages to secrete a series of cytokines that aided bone regeneration specifically [33]. However, only the correct duration of administration and the appropriate local concentration of Mg^2+^ could help Mg^2+^ exert its biological properties [33–35]. Barbeck et al. created a bone-defect model on a rabbit skull. They found that the Mg-alloy membrane did not lead to higher bone regeneration than that in blank sites [16]. However, our previous study using a bone-defect model in the rat skull indicated that Mg-Zn-REE membranes could promote bone healing significantly [21]. The main reason for the controversy stated above is that the geometry of the material, anticorrosion treatment, and implant position in the body affect the degradation of Mg-alloys and local concentration of Mg^2+^ [36]. An inappropriate concentration of Mg^2+^ can inhibit the proliferation and migration of cells, and even affect the differentiation of bone marrow mesenchymal stem cells [34, 35]. Therefore, controlling the degradation rate and duration of use of MG to match the osteogenesis process is important. The fresh DM could only play a role of osteoconduction [37, 38] and would not affect the results related to MG.

The article "Feasibility and Efficacy of a Degradable Magnesium-Alloy GBR Membrane for Bone Augmentation in a Distal Bone-Defect Model in Beagle Dogs" was published in 2022. Journal: Bioinorg Chem Appl.

However, there are some shortcomings in MG that need to be improved. A significant difference was not found in the values of VBH, NBF, or BV/TV 6 months after surgery (Figure 5). Those findings suggest that MG could promote bone healing initially, but did not improve the bone-defect height more effectively than BG. One explanation for this phenomenon is that the degradation rate of MG was too fast, which led to early loss of its mechanical properties to maintain the osteogenesis space, which is the key point for vertical augmentation of bone [8]. MG is degraded readily from the stress-concentrated part [39], which results in the loss of mechanical support ability before its complete degradation. The remains of MG were not observed in micro-CT images or histology 3 months after surgery, which indicated that MG lost its mechanical support ability much earlier. The surface coating could delay the degradation of Mg-alloy, but the tiny cracks and exudation of REEs on the surface of the material might be the weak points of fluorination treatment (Figure 3). The degradation of a material will accelerate as soon as the surface coating is broken [40, 41]. Wang et al. reported that a surface crack might be related to hydrogen release during fluorination [28] and it is not repaired by increasing the duration of fluorination [30]. Another explanation for poor osteogenic effect of MG is that the degradation of Mg-alloy led to the increase of local osteoclasts and the resorption of bone. It just explains why the TRAP (+) in the group MG was always slightly higher than that in the group BG (Figures 6(d)–6(f)). Osteoclasts are derived from the fusion of macrophages [34]. The degradation of MG produced insoluble degradation products which recruited macrophages to phagocytose (Figure 7). The fusion of macrophages to form osteoclasts led to bone resorption and affected the osteogenic effect of MG. Besides, the degradation of Mg-alloy resulted in an extremely alkaline and increasing Mg^2+^ microenvironments [42], which would aggravate local inflammation and increase osteoclasts and bone resorption. This highlights the importance of the mutual adaptation of material degradation and tissue growth. In addition, the degree of adhesion between MG and the tooth root could affect bone healing in the group MG [4]. To achieve better osteogenesis, the degradation rate of MG should be adjusted further to adapt to bone regeneration. The mechanical support ability of MG should be maintained for ≥3 months even if the stress is concentrated at one site. Also, the shape of MG should be adapted more closely to the defect area.

The article "Feasibility and Efficacy of a Degradable Magnesium-Alloy GBR Membrane for Bone Augmentation in a Distal Bone-Defect Model in Beagle Dogs" was published in 2022. Journal: Bioinorg Chem Appl.

MG exhibited good biocompatibility in vivo. Serious complications did not occur during follow-up. Most surgical sites healed clinically and histologically, and the prevalence of infection was 12.5% in the group MG (2/16) and 6.25% (1/16) in the group BG (*P* > 0.05). Besides, the two infected sites were on the P2 sites of the same dog, which indicated that the occlusal trauma of biting the cage might be the main cause of infection. Another site in the group MG (1/16) was found to suffer wound dehiscence <1 after surgery. The irregular shape and stress concentration of MG might be the cause of infection [43], which should be optimized in the future. With regard to gas accumulation during MG degradation, subcutaneous emphysema was not observed clinically. However, histology revealed that some gas cavities covered fibrotic tissue in one site in the group MG-3 m. Some researchers have proposed that fibrosis can isolate gas from surrounding tissue and influence bone regeneration [44]. However, other scholars hold the opposite opinion; comparing the gas cavities with some bone-substitute materials revealed induction of similar slight fibrotic encapsulation without interference with bone healing [16, 45]. The latter conclusion is more in accordance with observations in our study. A gas cavity was not found by histology in the group MG-6 m. The degradation products of MG were in close contact with new bone, which demonstrated that MG and its degradation products did not interfere with the formation of new bone.

The article "Feasibility and Efficacy of a Degradable Magnesium-Alloy GBR Membrane for Bone Augmentation in a Distal Bone-Defect Model in Beagle Dogs" was published in 2022. Journal: Bioinorg Chem Appl.

MG-related elements can be degraded through the lymphatic circulation without causing toxic reactions. Mg-alloy is degraded *via* noncellular dissolution and phagocytosis [13]. Fluorinated Mg-alloy is not soluble in water and resorbed mainly *via* phagocytosis, which was slower than noncellular dissolution and make the MgF_2_ on the surface of MG enhance the corrosion resistance of the substrate [16]. Previously, we implanted Mg-alloy into the skull-bone defects of rats and analyzed the metabolism of this material in various organs (brain, heart, liver, spleen, lungs, kidneys, adrenal glands, submandibular lymph nodes). The content of all material-related elements was within the safe range, but REEs metabolized slowly and accumulated in submandibular lymph nodes [21]. However, a long-term study to ascertain the effect on the lymph nodes was not done. We monitored the concentrations of MG-related elements in the submandibular lymph nodes for a long time. The concentration of Y and Nd in the group MG was significantly higher than that in the group BG (*P* ≤ 0.017). However, according to histology, bleeding or necrosis were not observed in the group MG, and the concentration of Y and Nd remained within the safe range. The contents of REEs were reduced gradually in the group BG, indicating that REEs could be metabolized slowly through the lymphatic circulation (Figure 8). Some researchers postulate that REEs in MG (especially Y and Nd with low toxicity) would not induce local toxicity [46, 47]. Controlling the dose of implanted REEs and avoiding “burst release” of Mg-REEs alloys is crucial. Further study should focus on reducing REE accumulation in the lymphatic system.

The main limitation of our study was a lack of short-term observation to describe MG degradation. The follow-up period was designed according to the duration of bone healing in humans [48], which is much longer than that for MG degradation. Future studies should focus on regulation of the degradation rate of MG.

## 5. Conclusions

We applied for the first time a model of mandibular bone defects to explore the influence of MG upon bone healing. MG exhibited good biocompatibility in vivo without leading to subcutaneous emphysema or increasing the infection risk compared with the use of BG. MG had the potential for osteoinduction, and its osteogenic effect was not inferior to that of BG. The osteogenic effect of MG could be enhanced by improvements in Mg-alloy. Future studies should explore the degradation rate that aids adaptation to bone formation in the oral cavity.

The article "Feasibility and Efficacy of a Degradable Magnesium-Alloy GBR Membrane for Bone Augmentation in a Distal Bone-Defect Model in Beagle Dogs" was published in 2022. Journal: Bioinorg Chem Appl.

## Figures and Tables

**Figure 1:** Surgical procedure. (a) The mesial root of bilateral mandibular P2 and P4 underwent root canal treatment. (b) P2 and P4 were hemi-sected, and the distal roots were removed and processed to autologous fresh dentin matrix (DM). (c, d) The mesial and buccal bone walls of the extraction sockets were removed to create a two-wall bony defect of dimension 5 mm × 5 mm × 5 mm to simulate M2M-DBD. (e) MAR-Gide was designed according to the characteristics of M2M-DBD. Some holes were processed for fixation of Mg nails and nutritional supply. (f–h) After grafting the DM in the bone defect, MAR-Gide and Bio-Gide were covered on the surface according to the study design. MAR-Gide was fixed with Mg nails. (i) Flaps were closed after tension reduction. All surgical sites were protected with periodontal dressing materials.

**Figure 2:** Measurement of vertical bone height (VBH) by micro-CT. The VBH was recorded as the linear distance from the enamel-cementum junction to the bottom of the bone defect.

**Figure 3:** Surface (5000x magnification) and cross section (500x) of SEM images and EDS of coatings fabricated on MAR-Gide. (a–d) The coating on MAR-Gide is uniform. Some particles composed of rare-earth elements are partially scattered on the surface (red arrow). Cracks of width <0.2 *μ*m are distributed uniformly (blue triangle). (e, f) A fluorinated film of thickness ∼3 *μ*m (red arrow) on MAR-Gide is uniform.

**Figure 4:** XPS of coatings fabricated on MAR-Gide. (a) High-resolution Mg2p spectrum at the surface of fluoride-coated Mg showing center and FWHM values for MgF_2_ and Mg (OH)_2_. (b) Elemental composition of surface coatings.

**Figure 5:** Morphometry of bone defect area using micro-CT. (a) Trabecular volume/total volume of ROI (BV/TV). (b) Trabecular thickness (Tb. Th). (c) Trabecular number (Tb. N). (d) Trabecular separation (Tb. S). (e) Vertical bone height (VBH). (f) Average bone mineral density (BMD). ^*∗*^*P* < 0.05, ^*∗∗*^*P* < 0.01.

**Figure 6:** Quantitative histology of bone formation in the bone defect area. (a, b) Van Gieson's-stained sections of bilateral P2 sites in one beagle dog ((a) group MG-3 m, (b) group BG-3 m). New bone repair can be clearly observed in the group MG, whereas the defect area in the group BG is filled mostly with fibrous connective tissue (blue star). The blue triangle denotes the remaining mesial root. The blue dashed line denotes the level of the enamel-cementum junction. (c) Percent new bone formation (NBF) in different groups. (d, e) TRAP-stained sections in different groups ((d) group MG-3 m, (e) group BG-3 m). TRAP (+) cells are shown by a red arrow. (f) Average number of TRAP (+) cells in different groups under field of views at 200x magnification. ^*∗*^*P* < 0.05, ^*∗∗*^*P* < 0.01.

The article "Feasibility and Efficacy of a Degradable Magnesium-Alloy GBR Membrane for Bone Augmentation in a Distal Bone-Defect Model in Beagle Dogs" was published in 2022. Journal: Bioinorg Chem Appl.

**Figure 7:** Histology of MAR-Gide degradation. (a–d) “Island-shaped” new bone is formed accompanied with the degradation products of MAR-Gide. (a, c) 25x magnification; (b, d) 200x magnification. (e, f) Degradation particles of MAR-Gide are “swallowed up” by monocytes (400x magnification). (g, h) Gas cavities are found in only one section in the group MG-3 m, which are divided into compartments surrounded with fibrotic tissue.

**Figure 8:** Histology and MG-related elemental analysis of submandibular lymph nodes. (a, b) Lymph nodes in the group MG-6 m. (c, d) Lymph nodes in the group BG-6 m. Pathological changes (e.g., bleeding and local necrosis) were not found in either group. (e–h) Content of MG-related elements in different groups. ^*∗*^*P* < 0.05, ^*∗∗*^*P* < 0.01.

## Data Availability

The data are available on request from the corresponding author.
